# Construction and Screening of Fractional Library of *Salviae Miltiorrhizae* Radix et Rhizoma for the Rapid Identification of Active Compounds against Prostate Cancer

**DOI:** 10.1155/2022/9955834

**Published:** 2022-02-24

**Authors:** Qing-Mei Ye, Xiaozhen Ji, Bin Wang, Miao Yu, Jin Cai, Weinv Zeng, Weikang Chen, Fangxuan Han, Guolei Huang, Caijuan Zheng

**Affiliations:** ^1^Hainan General Hospital, Hainan Affiliated Hospital of Hainan Medical University, Haikou, Hainan 570311, China; ^2^Key Laboratory of Tropical Medicinal Plant Chemistry of Ministry of Education, College of Chemistry and Chemical Engineering, Hainan Normal University, Haikou, Hainan 571158, China; ^3^Key Laboratory of Tropical Medicinal Plant Chemistry of Hainan Province, College of Chemistry and Chemical Engineering, Hainan Normal University, Haikou, Hainan 571158, China

## Abstract

Efficient screening of anticancer agents is in urgent need to develop new drugs that combat malignant tumors and drug resistance. In this study, a combined strategy composed by solvent partition and HPLC fractionation was developed to generate an herbal fraction library of *Salviae Miltiorrhizae* Radix et Rhizoma to quickly and efficiently screen anticancer agents. All library entries are directed into 96 well plates which are well mapped with HPLC chromatograms. The cell proliferation assay revealed seven active subfractions. Then, the major active ten peaks in these subfractions were prepared and isolated by semipreparative HPLC, and their inhibitory activities against prostate cancer cells were then tested at the same concentration level, leading to the identification of several active compounds. In addition, the structures of compounds arucadiol (**2**), 15,16-dihydrotanshinone I (**4**), methyl tanshinonate (**5**), cryptanshinone (**7**), 1,2-dihydrotanshinquinone I (**9**), and tanshinone IIA (**10**) were characterized by mass spectrometry and X-ray crystallographic analysis, and they were confirmed to be active in suppressing prostate cancer cell proliferation at 7.5 or 15 *μ*g/mL, among which, the minor compounds **2**, **4**, and **5** showed higher activities than **9** and **10**. This study provided a rapid strategy of identifying new anticancer agents in *Salviae Miltiorrhizae* Radix et Rhizoma, which can be applied in other herbal medicines.

## 1. Introduction

Herbal medicines, including certain extractions, or formulated traditional medicines, have been used for the treatment of various chronic and infectious diseases for thousands of years worldwide. Nowadays, they continue to play an important role in healthcare, and especially in new drug discoveries [1, 2]. It has been estimated by the World Health Organization that approximately 80% of the world's population use traditional medicines as their primary healthcare [3]. More importantly, approximately 30–40% of the approved drugs are derived from herbal medicine, further highlighting their critical role in drug discovery [4].

However, the active components of many herbs are still largely unknown. The chemical compositions, e.g., both in number and structures, in herbs tend to be very complex, since every herb usually contains hundreds or even thousands of phytochemicals (secondary metabolites), in addition to a large amount of proteins, polysaccharides, resins, and tannins (primary metabolite) which often undermine/impact the activity of the active components and usually lead to false positive effects [5–8]. Thus, a rapid isolation and screening system is in urgent need.

*Salviae Miltiorrhizae* Radix et Rhizoma (Danshen) is a typical example that contains complex chemical components and possesses multiple biological activities [9–11]. *Salviae Miltiorrhizae* Radix et Rhizoma, originally derived from the dry root of *Salvia miltiorrhiza*, is one of the most widely applied traditional herbal medicines in some Asian countries. This herb has been used extensively for the treatment of cancer, cardiovascular and cerebrovascular diseases, particularly in the angina pectoris and myocardial infarction [9, 12]. Besides the high content of polysaccharide, *Salviae Miltiorrhizae* Radix et Rhizoma contain two major groups of secondary metabolites, i.e., salvianolic acids and tanshinones [13, 14]. Growing evidence has indicated that the part of salvianolic acids is responsible for the cardiovascular and cerebrovascular tonic effects [15], while the tanshinones are found to show promising anticancer activities [16, 17], which is the focus of the current study. Growing evidence showed that tanshinone IIA induces apoptosis in human colon cancer Colo 205 cells through the downregulation of ErbB-2 (Erb-B2 receptor tyrosine kinase 2) protein expression and the upregulation of TNF-*α* (tumor necrosis factor-alpha) and caspase-3, a key player in regulating apoptosis [18]. Tanshinone IIA also exhibited strong inhibitory effects against human cervical cancer cells with an IC_50_ value of 8.49 *μ*M, and the proteomics study revealed that tanshinone IIA acted via the microtubule assembly pathway, leading to the G2/M phase arrest [19]. Similar effects were also validated in gastric cancer cells [20], esophageal carcinoma cells [21], and oral squamous cell carcinoma [22]. Another key component tanshinone I, significantly inhibited the migration, invasion, and gelatinase activity of non-small-cell lung cancer CL1-5 cells and also reduced the tumorigenesis and metastasis in CL1-5 cell xenograft mice [23]. While unlike tanshinone IIA, the mechanisms of the anticancer effects of tanshinone I were mediated through the modulation of IL-8 (interleukin-8), Ras-mitogen-activated protein kinase, and Rac1 signaling pathways [23, 24]. Tanshinone I also inhibited TNF-*α*-induced VEGF (vascular endothelial growth factor) production in breast cancer MDA-MB-231 cells and suppressed the migration of MDA-MB-231 cells through impacting extracellular matrix [25, 26]. In addition, another tanshinone, cryptotanshinone, was shown to inhibit prostate cancer DU145 cells through the inhibition of STAT3 (signal transducer and activator of transcription 3) [27].

By far, about fifty tanshinones were identified from *Salviae Miltiorrhizae* Radix et Rhizoma. However, only those tanshinones mentioned above were investigated as anticancer agents. In the current study, we attempted to unveil whether there are other active compounds in *Salviae Miltiorrhizae* Radix et Rhizoma that can inhibit prostate cancer cell growth. In order to rapidly and systematically identify antitumor components in *Salviae Miltiorrhizae* Radix et Rhizoma, it is necessary to develop an herbal fractional library that contains all the chemical components that possess sufficient purity for biological assays. Therefore, we developed a combined strategy composed with solvent partition and HPLC fractionation to generate the herbal fraction library of *Salviae Miltiorrhizae* Radix et Rhizoma. All library entries were then directed into 96-well plates which were well mapped with HPLC chromatograms. Accordingly, the proliferation suppressing activities were directly linked to the chemical profiles. We describe here the strategy and the library-based screening results for their anticancer potential.

## 2. Experimental

### 2.1. General Experimental Procedures

ESI-MS (electrospray ionization mass spectrometry) was recorded on a Finnigan TSQ 7000 mass spectrometer. Single crystal X-ray analysis was conducted on the Bruker Smart CCD 1000 diffractometer (Bruker, Billerica, MA, USA). An Agilent 1200 system was used to generate a fractional library. The Bionoon SpeedVac (Shanghai, China) was used to concentrate the subfractions from HPLC. HPLC-MS grade acetonitrile and methanol were purchased from Merck (Darmstadt, Germany), and MS grade formic acid from Sigma-Aldrich (Cat. No. 94318). Purified water was prepared in house with Millipore (Bedford, MA, USA). Other chemicals and solvents were of analytical grade. Column chromatography was performed with silica gel (Merck, Germany).

### 2.2. Extraction

The dried roots of *Salviae Miltiorrhizae* Radix et Rhizoma (1 kg) were extracted with MeOH (2500 mL) under ultrasonic conditions three times. Then, the extracted solutions were combined and condensed under reduced pressure to afford the crude extract.

### 2.3. Partition

The crude extract was suspended in distilled water and partitioned against ether and ethyl acetate to afford the ether (9.5 g), ethyl acetate (11.3 g), and water-soluble fractions (35.5 g), respectively.

### 2.4. Fractionation

Both the ether and ethyl acetate fractions were then dissolved in acetonitrile, and a stock solution (50 mg/mL) was prepared for each fraction. Then, each fraction was further divided into 20 subfractions by semipreparative HPLC as per the following conditions:

  Instrument: Waters 2695 with autosampler and the PDA detector.
  Mobile phases: A: H_2_O and B: acetonitrile (gradient: 0–20 min 20–30% B, 20–30 min 30–50% B, 30–40 min 50–70% B, 40–50 min 70–80% B, 50–60 min 80–80% B for the ether fraction). A: H_2_O and B: acetonitrile (gradient: 0–25 min 5–22% B, 25–50 min 22–30% B, 50–55 min 30–100% B, 55–57 min 100% B, 57–60 min 100–5% B for the ethyl acetate fraction and water-soluble fraction).
  Flow rate: 3 mL/min.
  Injection amount: 3 mg (50 mg/mL, 60 *μ*L).
  Collection rate: 3 min/fraction.

### 2.5. Library Construction

The forty HPLC subfractions from the ether fraction and the ethyl acetate fraction were concentrated by a Bionoon SpeedVac (Thermo Fisher Scientific, USA), and the residue was dissolved by 100 *μ*L of DMSO.

### 2.6. Cell Growth Assay

PC3 and LNCaP cells were seeded at a density of 3000 and 5000 per well, respectively, in the 96-well plate for overnight before the treatment. Cell growth inhibition was determined by the MTS proliferation kit (Promega) after 72 hours of treatment.

### 2.7. Semipreparative HPLC

The cell growth assay revealed several bioactive peaks. Then, semipreparative HPLC was used to directly purify those peaks from the mixture. The same HPLC conditions as described in the fractionation section were used.

### 2.8. Mass Spectrometry

Mass spectrometry was performed on a Waters Q-TOF Premier (Micromass MS Technologies, Manchester, UK) mass spectrometer. The nebulization gas was set to 650 L/h at 300°C, the cone gas was set to 50 L/h, and the source temperature was set to 80°C. The capillary voltage and sample cone voltage were set to 2700 V and 35 V, respectively. The Q-TOF Premier acquisition rate was set to 0.2 s with a 0.01 s interscan delay. Argon was employed as the collision gas at a pressure of 5.3 × 10^−5^ torr. The energy for collision-induced dissociation (CID) was set at 50%.

### 2.9. X-Ray Crystallography

The data collection was performed on a SMART 1000 CCD using graphite monochromated radiation (*λ* = 0.71073 Å). The structures were solved by direct methods (SHELXTL version 5.1) and refined by full-matrix least-squares on *F*^2^. In the structure refinements, nonhydrogen atoms were refined anisotropically. Hydrogen atoms were placed on the geometrically ideal positions by the ‘ride on' method [28, 29].

### 2.10. Statistics

The results in this study were presented and analyzed using the one-way ANOVA test by GraphPad. A *p* value less than 0.05 was considered to be significant.

## 3. Results

### 3.1. Generation of Bioactivity Chromatogram

To rapidly identify the active components that can inhibit prostate cancer cell growth, *Salviae Miltiorrhizae* Radix et Rhizoma was extracted with methanol, and the crude extract was divided into three fractions: ether, ethyl acetate, and water soluble. Both the ether (3 mg) and ethyl acetate fractions (3 mg) were further divided into twenty subfractions by semipreparative HPLC in 60 min. The subfractions were then dried by SpeedVac (Bionoon) and the residues were dissolved with 100 *μ*L of DMSO. Then, 3 *μ*L of each subfraction was used to first treat the PC3 cells. The distribution of inhibitory activities across the subfractions was revealed by the MTS assay. The correlation of the activity data with the well position (each well is equivalent to a 3 min fragment of the HPLC) allows the generation of a HPLC-bioactivity profile (Figure 1). Under this HPLC condition, the collection speed is 3 min per well, which corresponds to one or two peaks in the HPLC chromatograms, allowing the rapid characterization of these bioactive peaks.

### 3.2. Identification of Active Fraction and the Separation of Each Component

The cell growth assay revealed that fractions 14–20 in the ether soluble part and fraction EA17 in the ethyl acetate part showed about 60% inhibition against the PC3 cells. EA17, a profound peak in the HPLC profile, was identified as salvianolic acid B by MS analysis (C_36_H_30_O_16_, ESIMS, *m/z* = 717 [M-H]^−^); however, it was found to be inactive with no obvious inhibition against both PC3 cells at 50 *μ*M in the later validation test (Figure 2). Thus, the inhibitory activity of fraction EA17 might be attributed to the high concentration in the subfraction (which was >50 *μ*M). Accordingly, fractions of ether 14–20 were considered as active fractions. Then, semipreparative HPLC was used to directly purify the major peaks from each fraction. The collected solutions of these peaks were condensed by a rotary evaporator to afford compounds **1** (4.3 mg), **2** (3.2 mg), **3** (3.6 mg), **4** (5.8 mg), **5** (9.4 mg), **6** (6.6 mg), **7** (7.3 mg), **8** (4.1 mg), **9** (7.5 mg), and **10** (8.4 mg) from the seven fractions, respectively.

### 3.3. Compounds 2, 4, and 5 Showed Promising Anticancer Activities

In order to test if these compounds were really potent, their inhibitory activities were compared with those of untreated compounds under the same concentration of 7.5 and 15 *μ*g/mL in both PC3 and LNCaP cells, respectively. At 7.5 *μ*g/mL, compound **2**, **4**, **5**, and **7** showed 88.0%, 97.4%, 95.6%, and 86.4% inhibition against PC3 cells, and 93.2%, 96.1%, 95.0%, and 40.1% inhibition against LNCaP cells, respectively. None of other compounds at 7.5 *μ*g/mL exhibited over 50% inhibition against these two cell lines. However, when the concentration was increased to 15.0 *μ*g/mL, compounds **9** and **10** showed 34.5% and 47.3% inhibition against the PC3 cells, and 88.7 and 86.0% inhibition against the LNCaP cells, respectively (Figure 3).

### 3.4. The Crystal Structures of Active Compounds

To identify the structures of the active compounds **2**, **4**, **5**, **7**, **9**, and **10**, 2 *μ*L of each pure sample was subjected to HRMS (high resolution mass spectrometry) analysis. These structures were identified based on high resolution molecular ions, retention time, and UV spectra. Similarly, the other four nonactive compounds **1**, **3**, **6**, and **8** were also tested. The identification was carried out by comparison with the literature [30, 31], as shown in Table 1.

The abundant samples **7**, **9**, and **10** were then recrystallized in a mixture of hexane and ethyl acetate to afford red crystals, and their structures were further confirmed by single crystal X-ray analysis (Figure 4). Compounds **7**, **9**, and **10** shared the same carbon skeleton that was furan fused naphthoquinone. These compounds differed to each other by the positions of the double bonds and the substituent pattern. Compound **9** has one more double bond in ring A but only one methyl group at C-4 as compared with **7** and **10**. Rings B and C were in coplanar in all the three potent compounds. Ring D in compound **7** existed in an envelope conformation as compared with the coplanar conformation with rings B and C in **9** and **10** (Table 2).

## 4. Discussion

Traditional herbal medicines have been used for thousands of years in the world and serve as a rich source of bioactive lead compounds for new drug development [1, 4, 32]. Since each herb contains hundreds of or even thousands of chemical components [32], and the critical active components are often unknown, thus, it is imperative to identify the major and active components by well-designed and innovative isolation protocols and consequently, conduct the pharmacological study to disclose their therapeutic value [33]. Traditional isolation or separation of lead compounds from herbs followed by the bioassay guidance has long been used for the discovery of bioactive compounds [34]; however, it is often time-consuming and inefficient [35]. With the development of combinatorial chemistry and bioassay techniques simultaneously, high throughput screening based on the combinatorial strategies will become increasingly popular and more efficient [36]. We hypothesized that the complex chemical components in herbs can be considered as a natural combinatorial library that could be separated and grouped into different fractions through column chromatography. Compared to the synthetic chemical library that always contains compounds of the same type, this natural fractional library possesses abundant chemical diversities and is inexpensive and easily made. Our current investigation proposed a novel approach to construct and screen herbal fraction library for the rapid identification of active anticancer compounds, through which a direct link between the bioactivity (anticancer) profiles and the corresponding chemical profile of crude extracts will be achieved. The success of such approach would facilitate the decisions to be made for the subsequent purification steps and the further anticancer efficacies validation.

Our current investigation showed that a combination of HPLC and cell-based assay is a feasible strategy in rapidly screening active components in *Salviae Miltiorrhizae* Radix et Rhizoma. The results also showed that the minor compounds **2**, **4**, and **5** were more potent in suppressing prostate cancer cell growth than those of **7** and **10** which were the major components. Our future direction will focus on the anticancer potencies of these active compounds in different cancer types and cells, and unveil the mechanisms. Furthermore, these active compounds identified in this work can also serve as candidates for new anticancer agents, as well as lead compounds for further structural modification.

## Figures and Tables

**Figure 1:** Structural formulae of the ten components identified from *Salviae Miltiorrhizae* Radix et Rhizoma.

**Figure 2:** Bioactivity profiles of the subfractions from the ether fraction and ethyl acetate fractions of *Salviae Miltiorrhizae* Radix et Rhizoma. A variance of *p* value was calculated using the one-way ANOVA test. The differences compared with the vehicle control at the levels of ^*∗*^*p* < 0.05, ^*∗∗*^*p* < 0.01, and ^*∗∗∗*^*p* < 0.001 were considered statistically significant.

**Figure 3:** Inhibition of PC3 and LNCaP cells by compounds **1**–**10** at the concentrations at 7.5 and 15 *μ*g/mL. A variance of *p* values obtained was calculated using the one-way ANOVA test. The differences compared with the vehicle control at the levels of ^*∗*^*p* < 0.05, ^*∗∗*^*p* < 0.01, and ^*∗∗∗*^*p* < 0.001 were considered statistically significant. Taxol was used as the positive control (the cell viabilities were 1.5% and 2.4% for PC3 cells and 1.3% and 2.1% for LNCaP cells at the concentrations of 7.5 and 15.0 *μ*g/mL, respectively).

**Figure 4:** The structures of compounds **7**, **9**, and **10** as determined by X-ray diffraction.

**Table 1:** Characterization of tanshinones in Danshen by HPLC and mass spectrometry.

Compounds	RT	[M+H]^+^	UV max	Identification^*∗*^
**1**	39.3	297.1392	264	Danshenxinkun A
**2**	42.2	299.1479	225	Arucadiol
**3**	45.2	295.1224	262	3*α*-Hydroxymethylenetanshinone
**4**	46.3	279.0953	244	15,16-Dihydrotanshinone I
**5**	46.5	339.1246	225,268	Methyl tanshinonate
**6**	47.1	281.1169	245	Trijuganone B
**7**	48.0	297.1392	264	Cryptanshinone
**8**	51.9	277.0805	272	Tanshinone I
**9**	54.8	279.1020	290	1,2-Dihydrotanshinquinone I
**10**	59.2	295.1524	268	Tanshinone IIA

Note: ^*∗*^the data were in consistent with published data (Journal of Organic Chemistry 1990, 55(11), 3537–43 and Rapid Communications in Mass Spectrometry (2006), 20(8), 1266–1280).

**Table 2:** Crystal data and structure refinement for compounds **7**, **9**, and **10**.

Compound	7	9	10
CCDC deposit no.			
Color/shape	Red/block	Red/block	Red/block
Cryst dimens, mm^3^	0.56 0.34 0.20	0.50 0.36 0.25	0.58 0.37 0.15
Chemical formula	C_19_H_20_O_3_	C_18_H_14_O_3_	C_19_H_18_O_3_
Formula weight	296.35	278.29	294.34
Temperature, K	293 (2)	293 (2)	293 (2)
Crystal system	Orthorhombic	Triclinic	Orthorhombic
Space group	*P*2_1_2_1_2	*P*-1	*P*mna
Unit cell dimension	*a* = 14.466(1) Å	*a* = 8.693(2)Å	*a* = 6.701(1) Å
	*b* = 21.358(2) Å	*b* = 11.811(3)Å	*b* = 9.195(1) Å
	*c* = 9.8646(9) Å	*c* = 13.808(3)Å	*c* = 24.466(4) Å
		= 98.32(1)	
		= 95.31(1)	
		= 103.33(1)	
Volume, Å^3^	3047.8(5)	1353.3(5)	1507.7(5)
*Z*	8	4	4
Density, Mg/m^3^	1.292	1.366	1.297
Abs coeff, mm^−1^	0.086	0.093	0.087
Diffractometer/scan	Bruker CCD	Bruker CCD	Bruker CCD
Range, deg	1.70 to 25.02	1.50 to 25.12	1.66 to 24.99
Reflections mesd	16492	7399	7877
Indepnt reflns (*R*_int_)	5381 (0.0371)	4766 (0.0347)	1449 (0.1026)
Obsd reflns [*I* > 2*I*]	3788	2239	973
Data/params	5381/383	4766/379	1449/136
Extinction coeff	0.0018(5)	0.000	0.000
Goodness of fit on *F*^*2*^	1.054	0.894	1.021
*R*_1_ [*I* > 2(*I*)]	0.0614	0.0453	0.0550
*wR*_2_ (all data)	0.0907	0.1177	0.0827

*R*_1_ = ||*F*_o_| − |*F*_c_|| |*F*_o_|, *wR*_2_ = [ [*w*(*F*_0_^2^ − *F*_*c*_^2^)^2^] [*w*(*F*_0_^2^)^2^]]^1/2^.

## Data Availability

The data used to support the findings of this study are available from the corresponding author upon request.
